# A Case Series of Paederus Dermatitis: Understanding Its Varied and Diverse Clinical Presentations

**DOI:** 10.7759/cureus.54148

**Published:** 2024-02-13

**Authors:** Bhanupriya Tamilselvan, Srikanth Shanmugam, Pragasam Shakthi

**Affiliations:** 1 Dermatology, Mahatma Gandhi Medical College and Research Institute, Puducherry, IND

**Keywords:** burning sensation, blister beetle dermatitis, nairobi eye, vesiculobullous skin lesions, dermatitis linearis, kissing lesions, paederus dermatitis, irritant contact dermatitis (icd), rove beetles, blister beetle

## Abstract

Introduction

*Paederus* dermatitis arises from inadvertent skin contact with insects of the genus *Paederus*, leading to irritant contact dermatitis. This study aims to highlight the diverse clinical presentations and the remarkable ability of the disease to mimic various dermatological conditions.

Methodology

A total of 15 patients diagnosed with *Paederus* dermatitis in a period of four months from August 2023 to November 2023 were included in this retrospective study. The demographic profile, detailed history, clinical presentation, and site of lesion distribution were documented.

Results

Out of 15 patients, nine were males, and eight were females. All patients exhibited a sudden onset of lesions accompanied by burning and pain, with an average duration of approximately 2.5 days. The most prevalent clinical presentation was the linear type, followed by kissing lesions, an erythematous patch with a central gray area, Nairobi eye, burnt appearance, and post-inflammatory pigmentation.

Conclusion

*Paederus* dermatitis is common in tropical areas like India but is prone to misdiagnosis due to its varied presentation. Increased awareness can lead to accurate diagnoses and simpler treatment plans, reducing patient confusion.

## Introduction

*Paederus* dermatitis is an irritant contact dermatitis caused by the accidental crushing of rove beetles, which releases a vesicant chemical, pederin. Contact of the skin with this potent blistering chemical through crushing results in the sudden onset of erythematous skin with vesicles and bullae with severe burning and stinging. The vesicant pederin is predominantly released at toxic doses by female rove beetles that bear endosymbiotic bacteria *Pseudomonas* species [1]. This beetle does not bite or sting, but accidental crushing or brushing against the skin causes the release of its hemolymph containing pederin that causes painful necrotic blisters [2-4].

## Materials and methods

A retrospective case series analysis study was done in the Dermatology Department of Mahatma Gandhi Medical College and Research Institute located in Puducherry, India, for four months between August and November 2023. Approval for the said study was obtained from the Institutional Human Ethics Committee of Mahatma Gandhi Medical College and Research Institute (approval number: 314). All the patients who had attended the Dermatology Outpatient Department (OPD) during the study period with a clinical diagnosis of *Paederus* dermatitis made by the consultant were included. A total of 15 patients were included in the study, and all the clinical data was retrieved from the patient management system at the hospital. A detailed sociodemographic and clinical history included age, gender, patient's residential area, patient's awareness of any insect contact, sudden onset of lesions after waking up/travel, clinical morphology of the lesions, site of lesion, and associated symptoms such as burning, pain, blisters, or scarring. A case study proforma was made bearing all the relevant details. All these details were documented in the case study sheet. Data analysis was done using IBM SPSS Statistics for Windows, Version 22.0 (Released 2013; IBM Corp., Armonk, New York, United States), and results were expressed in frequency and percentage.

## Results

In this case series study of 15 patients, the gender distribution was nine male and eight female patients. The clinicodemographic details of all the patients included in the study were recorded (Table 1). Thirteen patients recognized the onset of lesions post-sleep cycle, while two out of 15 patients did not correlate it with sleep or travel. Only two patients had prior knowledge of insect contact preceding the onset of lesions, and both of them noticed it during travel in a bus with the windshield open.

**Table 1:** Clinicodemographic details of the patients included in the study

Patient	Sex	Age (years)	Locality	Knowledge of contact with insect	Proximity to field or terrestrial areas	Onset of lesions after sleep/travel
1	Male	60	Rural	No	Yes	Yes
2	Male	43	Rural	No	Yes	Yes
3	Male	10	Rural	No	Yes	Yes
4	Female	35	Rural	No	Yes	No
5	Female	42	Urban	Yes	No	Yes
6	Male	28	Urban	No	Yes	No
7	Male	36	Rural	No	Yes	Yes
8	Female	12	Rural	No	Yes	Yes
9	Male	29	Urban	No	Yes	Yes
10	Male	33	Rural	No	Yes	No
11	Female	45	Rural	No	Yes	Yes
12	Male	52	Rural	No	Yes	Yes
13	Female	50	Rural	No	Yes	Yes
14	Female	47	Rural	No	Yes	Yes
15	Male	46	Rural	Yes	No	Yes

Regarding symptom presentation, burning was uniformly reported in 14 out of 15 patients (93.3%) with active lesions, redness in 14 out of 15 patients (93.3%), and blistering in 10 out of 15 patients (66.6%), and pain was observed in 12 out of 15 patients (80%). Only one patient presented late after the healing of the acute dermatitis with no symptoms. Additionally, severe wincing pain upon touch was noted in 14 out of 15 patients, corresponding to approximately 93.3% of the study group. The video demonstrating the pain on touching the lesion is given below (Video 1).

**Video 1:** Video demonstrating severe wincing pain on touching the lesion in Paederus dermatitis

Among the various morphological patterns observed, the predominant pattern was a linear erythematous plaque with vesicles (Figures 1A-1C). This linear pattern of presentation was identified in seven out of 15 patients (46.6%). This was followed by the next common pattern in our study which was erythematous lesions with a central gray area (Figure 2) which was observed in three patients contributing to 20% and kissing lesions (Figure 3) seen in two patients contributing to 13.3% of the study.

**Figure 1:** Linear presentation of blister beetle dermatitis over the left shoulder (A), left side of the neck (B), and right forearm (C)

**Figure 2:** Erythematous lesion with central gray area and peripheral vesicles over the right shoulder and lateral chest wall

**Figure 3:** Kissing lesion over the right cubital flexural area

A burnt appearance of the skin (Figure 4) was noted in one patient contributing to 6.6% of the study. Other patterns noted were Nairobi eye appearance (1% in one patient) and post-inflammatory hyperpigmentation (6.6% in one patient), respectively. All the patterns of clinical presentation and associated symptoms at presentation are summarized in Table 2.

**Figure 4:** Burnt appearance over the left side of the neck

**Table 2:** Symptom presentation and morphological patterns of Paederus dermatitis

Variables	Number	Percent
Symptoms		
Pain	12	80%
Redness	14	81%
Blistering	10	66.6%
Burning	14	93.3%
Severe pain on touch	14	93.3%
Morphology		
Linear lesion	7	46.6%
Kissing lesion	2	13.3%
Erythematous lesion with gray area	3	20%
Burnt appearance	1	6.6%
Nairobi eye	1	6.6%
Post-inflammatory hyperpigmentation	1	6.6%

The average duration of the lesion lasted from two to 10 days in all patients. All lesions were present only on the exposed area of the body with the face and neck as the commonest sites in nine of 15 patients, followed by the trunk and upper limbs in three patients each. 

## Discussion

*Paederus* dermatitis, also known as "dermatitis linearis," "rove beetle dermatitis," and "Staphylinidae dermatitis," is caused by beetles of the order Coleoptera, genus *Paederus*, under subfamilies Meloidae, Oedemeridae, and Staphylinidae. *Paederus* dermatitis is known to be an entomological model of irritant contact dermatitis [2-5]. Sometimes, *Paederus* dermatitis is referred to as blister beetle dermatitis. But it should be noted that *Paederus* dermatitis is caused by beetles of the Staphylinidae family of the order Coleoptera and blister beetle dermatitis is caused by the beetles of Meloidae and Oedemeridae families of the order Coleoptera. Pederin, the toxin responsible for *Paederus* dermatitis, is produced by endosymbiotic *Pseudomonas* bacteria within *Paederus* beetles. Blister beetle dermatitis also known as cantharidin dermatitis is caused by the toxin cantharidin. Non-inflammatory vesicles and bullae characterized it. Cantharidin has a different chemical structure from pederin and induces a less cutaneous violent reaction that occurs within a few hours of exposure [6,7].

Reaction to pederin has a delayed onset, typically occurring 12-48 hours post exposure. Scarring and hyperpigmentation are commonly observed after *Paederus* dermatitis, whereas dermatitis from cantharidin rarely results in scarring. *Paederus* dermatitis is characterized by vesicles, bullae, and pustules arising on intensely inflamed skin. Acute dermatitis caused by pederin occurs corresponding to the shape and dimension of the area over which the vesicant chemical was released. *Paederus* dermatitis is a self-healing condition [6,8-11].

The breakout in the number of cases has been often noticed to occur during or after rainy seasons [3,11-18]. Adults of a few *Paederus* species are at times very abundant, especially in tropical countries [15]. *Paederus* beetles, notably *Paederus melampus*, are associated with dermatitis outbreaks in countries like Sri Lanka and India, with high prevalence in regions of India such as Odisha, West Bengal, Punjab, Rajasthan, and Tamil Nadu and Karnataka. These beetles, typically measuring 7-10 mm in length, inhabit moist environments, feeding on small insects and plant debris. Various species of the genus *Paederus*, found globally, are primarily nocturnal and are strongly attracted to light. In our study, 14 out of 15 patients reported noticing lesions immediately upon waking from sleep, aligning with the nocturnal activity of the beetle. While they typically do not bite or sting, their hemolymph, when crushed on contact, acts as a potent irritant, causing irritant contact dermatitis [3]. If the beetles are found on the skin, brushing them off, rather than crushing them, avoids producing dermatitis [17].

The predominant symptoms reported were pain, itching, redness, and tenderness in exposed parts of the body. This finding is similar to the other findings reported in other studies, by Kellner and Dettner [10] and Gyeltshen et al. [11]. The majority of the lesions presented were linear erythematous followed by erythematous lesions with gray centers. The mean duration of the skin rash from onset until recovery was 13 days. Our study findings were similar to studies done by Gyeltshen et al. [11]. 

Most people are unaware of contact with the insect as it usually occurs at night during sleep when the insects are crushed reflexly. Dermatitis caused by *Paederus* affects individuals of any gender, age, race, or social background, depending on their activities and the presence of insects. The condition is more commonly observed in exposed areas of the skin. The incidence of cases tends to be higher in the last quarter of the year, following the rainy season [3,17]. Symptoms manifest within 24-48 hours after contact and may take a week or more to resolve. Mostly exposed areas of the body are affected. The characteristic linear appearance of this lesion is due to the crushing of the insect and the subsequent smearing of the toxin on the skin. A drip mark is occasionally seen when the toxin has run down the skin producing whiplash dermatitis [12]. These findings in a study by Karthikeyan and Kumar were similar to our study [6]. 

The lesions are characterized by erythema and edema, often appearing linear and resembling a whiplash. Vesicles typically emerge towards the center of the affected area, frequently progressing to pustules [5,8]. Complications of *Paederus* dermatitis encompass post-inflammatory hyperpigmentation, secondary infections, and severe exfoliating and ulcerating dermatitis that may necessitate hospitalization [5]. Additionally, conjunctivitis caused by pederin exposure is sometimes mistaken for preseptal cellulitis, an ocular infection [18-22].

Clinical presentations vary based on morphological types. Dermatitis linearis is the most common pattern and occurs in any exposed site. The characteristic presentation is erythematous vesicles and pustules with edema arranged in a linear pattern resembling a whiplash [6]. The localized pustular dermatosis pattern mimics irritant contact dermatitis, displaying grouped pustules at the insect-crushed site [6,14,16]. The other clinical pattern is an erythematous patch with an irregular border, which develops an increasingly gray, necrotic center, appearing similar to a burn. The pathognomonic lesions of *Paederus* dermatitis are kissing lesion patterns. This develops when damaged skin surfaces come into contact with previously unaffected skin, such as in the flexures of the elbow or adjacent surfaces of the thighs [6,14,17]. The uncommon but still reported variants of *Paederus* dermatitis include (a) extensive skin involvement with systemic symptoms like fever and vomiting, (b) genital lesions that arise from passive toxin transfer from other exposed areas of the skin, (c) Nairobi eye variant which is associated with ocular toxin involvement which may present as unilateral periorbital dermatitis with keratoconjunctivitis and the name originating from Zaire in 1915, (d) atypical presentation of *Paederus* dermatitis which presents as diffuse erythematous and desquamative lesions primarily on the upper body and face, (e) erythrodermic presentation involving more than 90% of body surface area with erythema and scaling, and (f) systemic involvement of the lung. Lymph nodes can also be seen very rarely in *Paederus* dermatitis [6,14,16,17,22-28]. The atypicality in clinical presentation can be attributed to the following factors: contact with specific *Paederus* species, repeated exposure in endemic areas, underlying immune disorders like atopy, immunological phenomena, and impact of infested water sources [29]. Systemic involvements requiring admissions are also reported in a study by Padhi et al. Vasculitis-like *Paederus* presentation, erythema multiforme-like presentation, and lung involvement have also been documented [2-4,30]. 

*Paederus* dermatitis is often confused with many dermatological diseases owing to the clinical similarities like herpes zoster and herpes simplex, bullous impetigo, pustular psoriasis, Sneddon-Wilkinson disease, fungal infections, and allergic reactions [12,16,22]. 

Considering the analysis of our case study and review of the literature on various *Paederus* dermatitis cases, we can clearly understand that the diagnosis of this dermatitis is strongly based on complete history-taking and careful clinical examination of the lesions. We have proposed a diagnostic aid system to confirm the diagnosis of *Paederus* dermatitis. The following data from history which includes (i) history of contact with any insect, (ii) onset of lesions noticed after sleep or travel, (iii) patient's locality, especially if surrounding a field or from an endemic region of *Paederus* dermatitis, (iv) objective criteria for diagnosis, (v) sudden onset of lesions, and (vi) presence of severe pain and burning sensation can be elicited to make a diagnosis. The presence of any of the morphological patterns like the most commonly seen linear or streaky pattern of dermatitis with or without kissing lesions and erythematous patches with central gray necrotic burn-like lesions can be noted. The correlation of data from history and clinical findings will lead to a most probable diagnosis of *Paederus* dermatitis. Since any dermatoses with vesiculobullous lesions can be put as a differential to *Paederus* dermatitis, a diagnostic checklist system as mentioned in our study can be useful in the appropriate diagnosis of the same. 

Limitations of the study

The smaller sample size was the limitation of the study.

## Conclusions

*Paederus* dermatitis is an acute condition caused by beetles mostly in tropical areas. Learning to recognize *Paederus* beetles and avoiding handling or crushing by blowing off these insects from the skin will help decrease these eruptions. Closing the doors and windows and turning off the light sources in sleeping areas can be practiced to help reduce contact with these insects. Clinical knowledge of various morphological patterns of *Paederus* dermatitis and correlating the salient points from the patient's history will enable the physician to flinch the correct diagnosis, not only improving the patient's treatment outcome but also preventing misdiagnosis. 
